The article "Controversy on Positive Peritoneal Cytology of Endometrial Carcinoma" was retracted in 2023. Reasons: unreliable results or conclusions; concerns about the data; concerns about the peer review; concerns about the citations.

# Controversy on Positive Peritoneal Cytology of Endometrial Carcinoma

**DOI:** 10.1155/2022/1906769

**Published:** 2022-04-01

**Authors:** Yi-Si Liu, Hui-Min Wang, Yan Gao

**Affiliations:** Department of Gynecology, Cancer Hospital of China Medical University, Liaoning Cancer Hospital & Institute, Shenyang, 110042 Liaoning, China

## Abstract

Endometrial carcinoma (EC) is one of the most common gynecological malignancies. Its incidence rate has been increasing year by year. The prognostic factors and treatment strategies of EC have aroused wide concern. The effects of peritoneal cytology on the prognosis and treatment of EC remain controversial. Some factors, such as differentiation degree, muscle invasion, and tumor size, are related to positive peritoneal cytology. Hysteroscopy is commonly used in the diagnosis and treatment of endometrial cancer, but hysteroscopic surgery may cause the tumor to spread into the abdominal cavity, resulting in positive peritoneal cytology. In this review, we discuss the factors related to positive peritoneal cytology and the influence of positive peritoneal cytology on the prognosis of endometrial cancer. Suspicious positive peritoneal cytology may be an independent risk factor for endometrial cancer. The positive rate of peritoneal tumor cells in type II endometrial cancer is higher than other cells and is an independent risk factor for type II endometrial cancer. We also discuss the effects of peritoneal cytology on treatment decisions. Aggressive treatments seem to be more beneficial for patients with positive ascites cytology, but there is a lack of large-scale prospective clinical studies on their effectiveness and safety. The application of peritoneal cytology for endometrial cancer has been decreased in recent years. We believe that peritoneal cytology is necessary for this type of cancer. However, more studies on peritoneal cytology in endometrial cancer should be carried out.

## 1. Introduction

Endometrial carcinoma is one of the most common gynecological malignancies. There are 319 500 new cases in the world every year, and the mortality is as high as 23% [1, 2]. The main risk factors for endometrial cancer include genetic correlation [2–4] (Lynch syndrome, Cowden syndrome, etc.), continuous estrogen stimulation, and metabolic syndrome. In recent years, with changes in diet and lifestyle, the incidence of endometrial cancer has been gradually increasing [5, 6]. At present, early screening of endometrial cancer has not been widely used. The diagnosis is made mainly by diagnostic curettage or hysteroscopic endometrial biopsy, and the preliminary clinical staging is carried out [7]. The treatment of endometrial cancer is mainly surgery and comprehensive treatment according to the patient's condition [8]. Targeted therapy and immunotherapy are also widely used for endometrial cancer [9, 10]. The prognosis of endometrial carcinoma is related to the age of onset, stage, degree of tumor differentiation, and pathological type [11–15].

The article "Controversy on Positive Peritoneal Cytology of Endometrial Carcinoma" was retracted in 2023. Reasons: unreliable results or conclusions; concerns about the data; concerns about the peer review; concerns about the citations.

According to the different etiology and prognosis of endometrial cancer, Bokhman [16] divided it in 1983 into type I hormone dependent with good prognosis and type II hormone independent with poor prognosis. The common histopathological types are endometrioid carcinoma, serous carcinoma, clear cell carcinoma, and undifferentiated carcinoma [17]. Clinical staging is based on the 8th edition of the American Joint Cancer Committee (2017 edition) staging and the International Federation of Gynecology and Obstetrics (FIGO) [18] staging (2009 edition). The main treatment for endometrial cancer is surgery and chemoradiotherapy. The prognostic factors of endometrial carcinoma include pathological type, tumor stage, age, molecular typing, and vascular invasion [19]. According to the Federation International of Gynecology and Obstetrics (FIGO) in 1988 [20], endometrial cancer with positive peritoneal cytology is classified as phase IIIA. It is suggested that positive peritoneal cytology is one of the high-risk factors affecting prognosis of endometrial cancer, although FIGO revised the staging criteria in 2009 [21], and positive peritoneal cytology was not included. National Comprehensive Cancer Network (NCCN) [22] guidelines for endometrial cancer and Japan Society of Gynecologic Oncology (JSGO) guidelines [23] still recommend that peritoneal cytology be retained. The effect of positive peritoneal cytology on prognosis is still controversial. We discuss the effect of positive peritoneal cytology on prognosis of endometrial cancer and the effect of hysteroscopy on peritoneal cytology.

## 2. Effect of Hysteroscopy on Peritoneal Cytology

The gold standard for the diagnosis of endometrial cancer is histopathological examination [24]. There are two main ways to obtain histopathological specimens: fractional curettage [25], a traditional diagnostic method; and the guidelines recommend hysteroscopy as the preferred diagnostic method. Diagnostic curettage is a necessary skill for gynecologists and obstetricians, and it is widely used in the diagnosis and treatment of abnormal vaginal bleeding. Diagnostic curettage [26] has the advantages of simple and easy operation and less trauma. It enables pathological examination of the uterine cavity and cervical canal, and hysteroscopy can be used to treat vaginal bleeding caused by endometrial lesions. Under the direct vision of hysteroscopy, the location of suspicious lesions can be observed closely, and the range of abnormal lesions and the degree of lesion invasion preliminarily judged. Due to its visual controllability and magnification effect, hysteroscopy is more accurate than diagnostic curettage in sampling both sides of the uterine angle and the lower uterine segment near the cervical canal. Garzetti et al. [27] and Zhu et al. [28] have proved that the pathological diagnosis rate and postoperative pathological coincidence rate of hysteroscopy are significantly higher than those of diagnostic curettage, and the pathological diagnosis rate of hysteroscopy is as high as 97%. Hysteroscopy is more advantageous for thin endometrial carcinoma (intimal thickness only 2–3 mm) [29]. Current domestic and foreign guidelines for the treatment of early endometrial cancer with fertility preservation are mainly recommend hysteroscopic evaluation and local lesion resection combined with progesterone treatment [30, 31]. However, hysteroscopy is completed by uterine dilation (normal saline, glucose, and mannitol) under pressure compared with diagnostic curettage. At present, there is a widespread controversy about whether hysteroscopy increases the positive rate of tumor cytology and has an impact on prognosis. Some studies [32] have suggested that the positive and suspicious positive rates of peritoneal cytology in endometrial carcinoma by hysteroscopy are significantly higher than that in diagnostic curettage. Cohort studies [33] have suggested that although hysteroscopy increases the risk of positive peritoneal cytology in early endometrial cancer, it has no significant effect on prognosis. Vilos et al.'s study [34] showed that the positive rate of peritoneal cytology increased by 30% in patients with serous endometrial carcinoma before hysteroscopy. However, there was no significant difference in progression-free survival (PFS) and overall survival (OS) after 66 months of follow-up. One study [35] has suggested that although tumor cells may migrate to the peritoneal cavity during hysteroscopy, this is only temporary and peritoneal cytology becomes negative after some time. Obermair et al. [36] believe that if hysteroscopy is used for too long or too many lesions are removed to obtain more pathological tissues, it can cause lung metastasis of tumor cells under high-pressure perfusion via the blood vessels. Therefore, hysteroscopy should be performed carefully in patients with suspected endometrial cancer. Some studies [37] have suggested that uterine dilatation at a pressure <70 mmHg can significantly reduce the movement of intrauterine fluid from the fallopian tube into the abdominal cavity. In summary, diagnostic curettage can be selected for patients with highly suspected endometrial cancer by imaging, especially when the lesion is clear. In the case of necessary hysteroscopy, soft mirror and fine mirror can be used. In addition, in the case of suspected malignancy, the pressure of dilatation must be controlled.

The article "Controversy on Positive Peritoneal Cytology of Endometrial Carcinoma" was retracted in 2023. Reasons: unreliable results or conclusions; concerns about the data; concerns about the peer review; concerns about the citations.

## 3. Factors Related to Positive Peritoneal Cytology

A meta-analysis [38] has suggested that for patients with surgical stage 1 early-stage endometrial cancer, the incidence of myometrial invasion ≥1/2 tended to be higher and 5-year progression-free survival was worse in the positive peritoneal cytology group than the negative peritoneal cytology group. A retrospective analysis of the SEER database [39] has shown that the higher the tumor stage, the higher the positive cytology and suspicious positive rates are. In stage IA endometrial cancer, if the tumor diameter is ≤2 cm, the positive rate of peritoneal cytology is only 4%; if the tumor diameter is >2 cm, the positive rate of peritoneal cytology is 10%. The positive rate of peritoneal cytology in endometrial adenocarcinoma is about 6.8%, while that of serous carcinoma is 23.4%. Therefore, positive peritoneal cytology in endometrial carcinoma is closely related to tumor pathological type, tumor size, depth of invasion, lymph node metastasis, and other poor prognostic factors. Studies in China [40] have suggested that the prognosis of early endometrial carcinoma with positive peritoneal cytology is worse, which may be related to undetected peritoneal metastasis or micrometastasis.

## 4. Effect of Positive Peritoneal Cytology on Prognosis of Endometrial Carcinoma

NCCN and JSGO guidelines recommend that peritoneal cytology specimens should be retained for endometrial cancer staging surgery. ESMO-ESGO-ESTRO [41] guidelines did not retain peritoneal cytology specimens for early endometrial cancer staging surgery. A retrospective study [29] of the SEER database in the USA in 2018 showed that the collection of peritoneal cytology has decreased by 44% since 2010. Daix et al. [42] suggested that the missed peritoneal cytology during hysterectomy was related to an increased risk of death in women with endometrial cancer. Peritoneal cytology results are negative, suspicious positive, or positive. The patients with stage I–III endometrial cancer who had peritoneal cytology results during hysterectomy in the USA from 2010 to 2016 were retrospectively analyzed [43]. The positive rate of cytology was 8.0%, and the suspicious positive rate was 1.7%. Compared with negative cytology, women in the suspicious peritoneal cytology group were younger. Peritoneal-cytology-negative, 5-year OS rate was 86.8%, suspicious cytology-positive rate was 77.8%, and cytology-positive rate was 66.5%. After controlling variables, suspicious positive peritoneal cytology was an independent risk factor for endometrial cancer. The 5-year PFS was 8.2% for negative peritoneal cytology, 16.8% for suspicious positive cytology, and 28.7% for positive cytology. Multivariate analysis showed [44] that suspicious positive peritoneal cytology was associated with an increased risk of endometrial cancer mortality and could predict mortality. In 2021, a retrospective study [45] for >20 years was conducted to analyze the effect of peritoneal cytology on the prognosis of type II endometrial cancer. The positive rate of peritoneal tumor cells in type II endometrial cancer was as high as 22%. The positive rate of peritoneal cytology in patients with recurrence was 27%, and the positive rate of peritoneal cytology without recurrence was 16%. Positive peritoneal tumor cells were an independent risk factor for type II endometrial cancer.

The article "Controversy on Positive Peritoneal Cytology of Endometrial Carcinoma" was retracted in 2023. Reasons: unreliable results or conclusions; concerns about the data; concerns about the peer review; concerns about the citations.

## 5. Effect of Peritoneal Cytology on Treatment Decisions

In 2009, FIGO revised the staging criteria for endometrial cancer. Positive peritoneal cancer cells were not included in the staging of endometrial cancer. At present, ESMO [46], NCCN, and FIGO [47] guidelines do not provide treatment guidance for patients with positive or suspected positive peritoneal cytology. However, some studies [48] have shown that for stage II/III endometrial cancer patients with positive peritoneal cytology, combined chemotherapy and radiotherapy can improve survival rate, but not in patients with negative peritoneal cytology. In addition, in type II [49] endometrioid carcinoma, patients with stage II-III and positive peritoneal cytology only received chemotherapy; and for the peritoneal cytology negative patients, the effect of combined treatment effect is better. Aggressive treatment seems to be more beneficial for patients with positive peritoneal cytology, but there is a lack of large-scale prospective clinical studies on its effectiveness and safety (Figure 1).

## 6. Summary

In recent years, because the available guidelines for endometrial cancer with positive peritoneal cytology did not provide clear treatment recommendations, the application of peritoneal cytology has been decreased [50]; we believe that peritoneal cytology collection is necessary. Hysteroscopy has irreplaceable advantages in the diagnosis and treatment of endometrial cancer, but it has a certain probability of positive peritoneal cytology and tumor proliferation, and a new type of safe endometrial lesion sampling should be developed. Positive peritoneal cytology is related to many adverse prognostic factors of endometrial cancer, which is consistent with the results of high recurrence rate and low survival rate of patients with positive peritoneal cytology. Especially in type II endometrial carcinoma, the peritoneal tumor cell positive rate is high, and long-term prognosis is poor. At present, the optimal treatment strategy for patients with positive and suspected peritoneal tumor cells is still uncertain, which needs to be confirmed by large sample studies or prospective multicenter controlled studies. However, the current research results show that more active treatment of patients with positive peritoneal cytology may benefit patients. More studies on peritoneal cytology in endometrial cancer should be carried out.

The article "Controversy on Positive Peritoneal Cytology of Endometrial Carcinoma" was retracted in 2023. Reasons: unreliable results or conclusions; concerns about the data; concerns about the peer review; concerns about the citations.

## Figures and Tables

**Figure 1:** Peritoneal cytology results.

## Data Availability

The data used to support the findings of this study are available from the corresponding author upon request.
